The article "Diffusion Tensor Imaging Features of Watershed Segmentation Algorithm for Analysis of the Relationship between Depression and Brain Nerve Function of Patients with End-Stage Renal Disease" was published in 2021. Journal: J Healthc Eng.

# Diffusion Tensor Imaging Features of Watershed Segmentation Algorithm for Analysis of the Relationship between Depression and Brain Nerve Function of Patients with End-Stage Renal Disease

**DOI:** 10.1155/2021/7036863

**Published:** 2021-10-25

**Authors:** Feng Zhu, Jiao Xu, Mei Yang, Haitao Chi

**Affiliations:** ^1^Department of Nephrology, Dalian University Affiliated Xinhua Hospital, Dalian 116021, Liaoning, China; ^2^Department of Liver Diseases, Dalian Sixth People's Hospital, Dalian 116001, Liaoning, China; ^3^Department of Neurology, Dalian University Affiliated Xinhua Hospital, Dalian 116021, Liaoning, China

## Abstract

The aim of this research was to explore the relationship between depression and brain nerve function in patients with end-stage renal disease (ESRD) and long-term maintenance hemodialysis (MHD) based on watershed segmentation algorithm using diffusion tensor imaging (DTI) technology. A total of 29 ESRD patients with depression who received MHD treatment in the hemodialysis center of hospital were included as the research subjects (case group). A total of 29 healthy volunteers were recruited as the control group, and a total of 29 ESRD patients with depression and brain lesions were recruited as the control group (HC group). Within 24 h after hemodialysis, the blood biochemical indexes were collected before this DTI examination. All participants completed the neuropsychological scale (MoCA, TMT A, DST, SAS, and SDS) test. The original DTI data of all subjects were collected and processed based on watershed segmentation algorithm, and the results of automatic segmentation according to the image were evaluated as DSC = 0.9446, MPA = 0.9352, and IOU = 0.8911. Finally, the average value of imaging brain neuropathy in patients with depression in the department of nephrology was obtained. The differences in neuropsychological scale scores (PSQI, MoCA, TMTA, DST, SAS, and SDS) between the two groups were statistically significant (*P* < 0.05). The differences of FA values in all the white matter partitions of Fu organs, except the cingulum of hippocampus (CgH) between the two groups, were statistically significant (*P* < 0.05). ESRD and DTI quantitative detection under the guidance of watershed segmentation algorithm in MHD patients showed that ESRD patients can be early identified, so as to carry out psychological nursing as soon as possible to reduce the occurrence of depression, and then protect the brain nerve to reduce brain neuropathy.

## 1. Introduction

End-stage renal disease (ESRD) [1] is a worldwide public health problem. It generally refers to the middle and late stages of various types of chronic kidney diseases and has a certain degree of similarity with the concept of uremia. However, there are still some differences in diagnostic criteria. Generally, ESRD can be diagnosed when the glomerular filtration rate is low to a certain standard. This standard is generally recognized as 15 mL (min.1.73 m^2^) as the standard line. When the chronic kidney disease reaches the fifth stage, it enters the ESRD. At this stage, with the further decline of renal function, toxins continue to accumulate in the body, which may cause various symptoms of uremia. Generally, it relies on continuous maintenance dialysis or looking for appropriate renal sources for transplantation replacement therapy [2, 3]. In the ESRD for a long time, a large number of toxins accumulated in the body may cause damage to multiple important organs in the body. The central nervous system is the most likely to be affected. The central nervous system may cause many complications after injury, such as cerebrovascular injury, behavioral cognitive impairment, brain atrophy, cerebral infarction, and depression. According to relevant data, about 60% of ESRD patients have cognitive impairment, so it is of great significance to diagnose and intervene the brain structure changes of renal disease patients as soon as possible [4, 5]. However, the exact pathogenesis of cognitive impairment in ESRD patients is still unclear. Diffusion tensor imaging (DTI) can quantitatively display the abnormal pathological changes of white matter microstructure [6], and tract-based spatial statistics (TBSS) is a more ideal imaging method for automatic and efficient evaluation of white matter fiber integrity [7].

The article "Diffusion Tensor Imaging Features of Watershed Segmentation Algorithm for Analysis of the Relationship between Depression and Brain Nerve Function of Patients with End-Stage Renal Disease" was published in 2021. Journal: J Healthc Eng.

Watershed algorithm is a kind of algorithm technology derived from geodesy topology. It has many advantages, and the logical ideas in the algorithm are easy to understand. Therefore, it is widely used in various fields. Now, it is mainly used in image segmentation [8, 9]. The gradient map of the image to be segmented is regarded as the topology in geodesy [10, 11]. Watershed algorithm is a kind of applied morphology in general. Its main idea is to analogize the selected target image to topography. The gray value of the image represents the altitude of the terrain, and the gray pixels in the image represent the valleys and peaks in the terrain. It is assumed that a hole is placed on each extreme point of the gray pixel, and the analogy model is put into the water. At this moment, the terrain and area formed by the process of water rising from the extreme point are basins. Different catchment basins in the image are about to converge, and the junction of its convergence becomes a watershed [12]. The watershed algorithm is a mathematical morphological method, which belongs to a region segmentation technology, and is an effective image segmentation method. In addition, it is featured with fast calculation speed and more accurate positioning, so it has many applications in the field of image analysis. Marking extraction in an image is a method of controlling oversegmentation. The minimum value area of the original gradient image is forcibly modified by the previously mentioned marking, and irrelevant minimum values in the original gradient image are shielded, showing very good segmentation effect. DTI is currently the only noninvasive examination method that can track white matter fiber tracts in vivo and effectively observe it. It can directly show the spatial relationship between acute cerebral infarction lesions and fiber tract, so as to judge the severity of brain injury. At this stage, there are relatively few studies on the watershed algorithm in MRI DTT imaging on depression and brain nerve function in patients with ESRD. Therefore, in this study, the watershed algorithm was adopted to the image processing network, the DTI technology was applied to image the patient's CST, and the DTI images of brain injury were collected to understand the sleep, anxiety, and depression of patients in time and develop treatment plans for the patient as soon as possible to improve prognosis, so as to provide help for clinical diagnosis and treatment.

The article "Diffusion Tensor Imaging Features of Watershed Segmentation Algorithm for Analysis of the Relationship between Depression and Brain Nerve Function of Patients with End-Stage Renal Disease" was published in 2021. Journal: J Healthc Eng.

## 2. Methods

### 2.1. Research Objects

Twenty-nine ESRD patients who underwent hemodialysis in the hemodialysis center of the department of nephrology at a tertiary hospital from October 2018 to November 2019 were enrolled as the case group. Twenty-nine local healthy volunteers matched with the case group in age, gender, years of education, anxiety, depression, and sleep quality scores were enrolled. All subjects were educated for ≥6 years and were right-handed (Figure 1).

### 2.2. Inclusion and Exclusion Criteria

The inclusion criteria were as follows: (1) patients diagnosed with ESRD, according to K/DOQI chronic kidney disease classification criteria; (2) patients who underwent regular dialysis for three months; (3) patients with no history of renal transplantation or acute renal failure; (4) patients without previous headless trauma, intracranial occupation, stroke, mental and neurological diseases, metabolic diseases, and other diseases that may affect the nervous system; (5) patients with no history of smoking, drug addiction, or alcoholism; and (6) patients without MRI contraindications. This study was a prospective study and was approved by the hospital ethics committee. All subjects signed informed consent. The participants' general demographic information, conducted neuropsychological tests and MR scans, and relevant blood biochemical indexes were collected.

The article "Diffusion Tensor Imaging Features of Watershed Segmentation Algorithm for Analysis of the Relationship between Depression and Brain Nerve Function of Patients with End-Stage Renal Disease" was published in 2021. Journal: J Healthc Eng.

The exclusion criteria were as follows: (1) patients with lesions >1.0 cm in the brain confirmed by clinical history and conventional MRI examination, such as cerebral hemorrhage, cerebral infarction, and brain tumors; (2) patients who cannot complete the neuropsychological scale test; and (3) patients with MRI contraindications.

### 2.3. Watershed Segmentation Algorithm

Watershed algorithm is a kind of algorithm technology derived from geodesic topology. It has many advantages, and the logical ideas in the algorithm are easy to understand. Therefore, it is widely used in various fields. Now, it is mainly used in image segmentation [13, 14]. By applying this method to the field of image segmentation, it has made a significant contribution to optimizing the segmentation effect of the image. With further research on the watershed algorithm, the mathematical morphology technology was added to the segmentation field. Therefore, the complexity of the watershed algorithm is gradually improved, and the effect of the segmentation image is further improved. In different scenes and fields, the label and segmentation of the target image are realized at different levels, and the outline of the label parts after segmentation is clear.

The basic definition of watershed algorithm is as follows: the two-dimensional image *N* to be segmented is selected to set the discrete value in the interval of [0, M]. The image is defined as a gray image, where *M* is a positive number, and the following conditions need to be met:

(1) $$\begin{array}{c} D_{N}\varepsilon R^{2}⟶\left\{0,1,\ldots ,M\right\}, \end{array}$$

(2) $$\begin{array}{c} F⟶N\left(F\right). \end{array}$$

Let *U* be a grid, which represents a subset of the set *R*^2^ × *R*^2^. Each grid has different names according to the number of grids contained in it.

**Definition 1 .**

Pixel set with height of *H* is selected from the selected image *N*.

(3) $$\begin{array}{c} T_{H}=\left\{F\in D|N\left(F\right)\leq H\right\}. \end{array}$$

*H* represents the threshold, and *n*_*A*_ (*α*, B) geodesic distance is used to represent the distance between two points. The selection of these two points needs to satisfy *a*, *b* ∈ *A*. If *B* ⊆ *A* appears, region *B* is divided into random *G* regions, and *G* regions are connected with each other, denoted as *B*_*i*_, where *i* = 1,...,*G*.

**Definition 2 .**

In set *A*, *B*_*i*_ divided into random regions is selected, and the solution equation of the influence region corresponding to this part is as follows:

(4) $$\begin{array}{c} {\text{NR}}_{A}\left(B_{i},B\right)=\left\{F\in A|\left(F,B_{i}\right)<N_{A}\left(F,\frac{B}{B_{i}}\right)\right\}. \end{array}$$

**Definition 3 .**

The article "Diffusion Tensor Imaging Features of Watershed Segmentation Algorithm for Analysis of the Relationship between Depression and Brain Nerve Function of Patients with End-Stage Renal Disease" was published in 2021. Journal: J Healthc Eng.

Connect *B* and *B*_*i*_ to form a collection NR_*A*_(B).

(5) $$\begin{array}{c} {\text{NR}}_{A}\left(B\right)=\overset{G}{\underset{i=1}{\cup }}iR_{A}\left(B_{i},B\right). \end{array}$$

**Definition 4 .**

In set *A*, the absolute complement SKIZ of NR_*A*_(*B*) is considered to be the skeleton affecting some regions.

(6) $$\begin{array}{c} {\text{SKIZ}}_{A}\left(B\right)=\frac{A}{NR_{A}\left(B\right)}. \end{array}$$

After the pixels in the foreground part are concentrated, the SKIZ is obtained, and the following equations are derived:

(7) $$\begin{array}{c} z_{h_{\min}}=\left\{F\in D|N\left(F\right)=h_{\min}\right\}=T_{h_{\min}}, \end{array}$$

(8) $$\begin{array}{c} z_{G+1}={\text{MIN}}_{h+1}\cup NR_{T_{h+1}}\left(z_{h}\right),\;h\in \left[h_{\text{min}}-h_{\text{max}}\right]. \end{array}$$

**Definition 5 .**

In *D*, the watershed region Wshed (*f*) is the absolute complement set corresponding to *z*_*h*_max__.

(9) $$\begin{array}{c} \text{Wshed}\left(\text{f}\right)=\frac{D}{Z_{h_{\max}}}. \end{array}$$

If there is a big difference in the gray value between the selected image and the target image background, then it is believed that the segmentation effect is better. If the difference between the both is not obvious, the phenomenon of “undersegmentation” easily appears. Therefore, the contrast of the image is enhanced to a certain extent, and the mathematical morphology technology is added into the segmentation field, so that the gray value between the selected image and the background of the target image is greatly different. Let ut (*x*, *y*) and *f* (*x*, *y*) denote the denoised image and the gray image, respectively, and carry out the top-cap transformation on *f* (*x*, *y*) to retain the region with large brightness in the original image. The top-hat transformation result is as follows:

(10) $$\begin{array}{c} h=f-\left(f\circ b\right). \end{array}$$

*b* represents the structural element. *f*∘*b* represents the opening operation of *b* to *f*. The bottom-cap transformation is performed on *f* (*x*, *y*) to save the dark details in the image. The bottom-cap transformation result is as follows:

(11) $$\begin{array}{c} j=\left(f•b\right)-f. \end{array}$$

*f*·*b* denotes closed operation *b* to *f*. *h* (*x*, *y*) and *j* (*x*, *y*) are added to get contrast enhanced gray image.

(12) $$\begin{array}{c} i\left(x,y\right)=h\left(x,y\right)+j\left(x,y\right). \end{array}$$

i ⊕ b and i Θ b represent the expansion operation and corrosion operation of *b* to *i*, respectively, and the gradient of morphological image is as follows:

(13) $$\begin{array}{c} g=\left(i⊕b\right)-\left(i\Theta b\right). \end{array}$$

The flowchart of improved watershed segmentation algorithm is shown in Figure 2.

The article "Diffusion Tensor Imaging Features of Watershed Segmentation Algorithm for Analysis of the Relationship between Depression and Brain Nerve Function of Patients with End-Stage Renal Disease" was published in 2021. Journal: J Healthc Eng.

### 2.4. Assessment of Depression

Center for Epidemiological Survey, Depression (CES-D) was used to evaluate depression. One-way analysis of variance (ANOVA) was used to compare the differences among the three groups in terms of age, years of education, neuropsychological scale score, and DTI parameters (FA, MD, AD, and RD values) between the two groups. CES-D was designed to evaluate the frequency of current depressive symptoms, focusing on depression emotion or mood. CES-D, also known as the self-rating depression scale of stream invocation, was prepared by Sirodff at the National Institutes of Mental Health in 1997, known as the center for epidemiological studies depression scale. It is widely used in the field of depression diagnosis and is used in the clinical screening of patients with depressive symptoms in order to further check and diagnose them. Some also used an individual emotional examination to assess the severity of depressive symptoms. Compared with other self-rating depression scales, CES-D focuses more on the individual emotional experience and less on the somatic symptoms in depression. The minimum score of depression was 0, and the maximum score was 60. Psychologists set the 16 points as the dividing point. Those who scored above 16 points belonged to the depressed group, and those who scored below 16 points belonged to the nondepressed group. Sixteen to twenty points indicated mild depression, 21–25 points indicated moderate depression, and 26–60 points indicated severe depression. The degree of depression is easily affected by mood and mental state, so the measurement results may be different at different times, which is normal.

### 2.5. Inspection Equipment

#### 2.5.1. DTI Examination

All subjects underwent examination and data acquisition using Siemens Verio 3.0T superconducting magnetic resonance imaging (Magnetom Verio 3.0T) and used 12-channel standard head coil. The specific process and DTI parameters were as follows. Single excitation white-spin plane echo sequence was used. Specific parameters are as follows: echo time (TE) = 86 ms, repeat time (TR) = 11908 ms, slice number (slice) = 65, slice thickness (ST) = 2 mm, matrix size (MS) = 128 x 128, field of view (FOV) = 244 mm × 244 mm, voxel size (VS) = 2 mm × 2 mm × 2 mm, diffusion weighted directions = 30, and *b* value = 0s/mm^2^, 1000s/ram^2^. The total examination time was 12 min and 56 s.

#### 2.5.2. Blood Biochemical Examination Information

Before this MRI examination and within 24 h after hemodialysis, the patient group was tested for the following clinical biochemical indicators: serum creatinine (Scr), blood urea nitrogen (BUN), blood kalium (K), blood calcium (Ca), and blood phosphorus (P).

The article "Diffusion Tensor Imaging Features of Watershed Segmentation Algorithm for Analysis of the Relationship between Depression and Brain Nerve Function of Patients with End-Stage Renal Disease" was published in 2021. Journal: J Healthc Eng.

#### 2.5.3. MRI Examination

The nuclear magnetic resonance (NMR) scanning equipment, 1.5 T HDC nuclear magnetic superconducting magnetic resonance scanner of the United States, with 8-channel head coil, was used. The patients were allowed to maintain supine posture on the check bed. The head and neck joint coil was used to fix the head of the patients. The quality of the head coil was tested before routine scanning to ensure that the 12 channels of the coil were all working properly. Subjects wore earplugs to avoid excessive noise affecting the tester' s state, and then, all the MRI scan lights were turned off to avoid unnecessary light interference.

### 2.6. Statistical Method

SPSS19.0 software was used for statistical analysis. Measurement data conforming to normal distribution were expressed as mean ± standard deviation, and the difference between groups was analyzed by independent sample *t*-test. The measurement data that did not conform to the normal distribution were represented by median and quarter position, and the difference between groups was analyzed by nonparametric rank sum test. Count data were expressed as *n* (%). Differences between groups were analyzed by chi-square test. Pearson correlation analysis was performed for DTI diffusion index, depression score, and clinical biochemical index. *P* < 0.05 was considered statistically significant.

## 3. Results

### 3.1. Correlation Analysis of DTI Diffusion Indexes with Depression Score and Clinical Biochemical Indexes Based on Segmentation Algorithm

The correlation analysis in this study showed that the FA value in the anterior part of the left corona was positively correlated with the DST score (*r* = 0.586, *P*=0.007). The FA value of the right hook was positively correlated with MoCA score and negatively correlated with TMTA (*r* = 0.545, *P*=0.013; *r* = .0.464, *P*=0.039). Left Nd and subiculum MD values were negatively correlated with depression score (*r* = −0.463, *P*=0.040). There was no correlation between the values of FA, MD, AD, and RD in all the different brain regions and PSQI scores (*P* > 0.05). In addition, there was no significant correlation between the results of DTI dispersion indexes and the blood biochemical indexes of the subjects (*P* > 0.05) (Figure 3).

The segmentation results of the target image based on the watershed algorithm model are shown in Figure 4. The results of automatic segmentation based on the image were evaluated as DSC = 0.9152, MPA = 0.9229, and IOU = 0.8450. In order to improve the segmentation accuracy of the watershed model, the watershed algorithm with fine-tuning weight was tested to segment the target image. The image was processed independently under the algorithm processing, but the processing results were continuous and stable in time. The results are shown in Figure 4. The evaluation of the automatic segmentation results based on the image was DSC = 0.9446, MPA = 0.9352, and IOU = 0.8911.

The article "Diffusion Tensor Imaging Features of Watershed Segmentation Algorithm for Analysis of the Relationship between Depression and Brain Nerve Function of Patients with End-Stage Renal Disease" was published in 2021. Journal: J Healthc Eng.

### 3.2. Comparison of Neuropsychological Cognitive Scores among Subjects

The differences in MoCA score and TMT_A score between the ESRD group and the HC group were statistically significant (Figure 5).

### 3.3. Comparison of Difference Values in DIC Measurement of Brain Volume by ESRD

Compared with the HC group, almost all white matter areas of ESRD maintenance hemodialysis patients had decreased FA value and increased MD value and RD value. Only in the right superior corona radiata, left superior corona radiata, right superior longitudinal bundle, the difference was statistically significant (*P* < 0.05) (Figure 6).

### 3.4. Comparison of General Condition between Depression Group and Nondepression Group

A total of 176 questionnaires were distributed to patients with regular hemodialysis for more than half a year in the hemodialysis room and were distributed and recovered by the competent nurses in the dialysis room. The recovery rate was 100%. There were 103 males and 73 females, with an average age of 61.24 ± 12.08 years. There were 58 cases in depression group and 29 cases in nondepression group. The number of depression accounts for 66% of the total. The general status of the two groups was significantly different in personal monthly income and working status (*P* > 0.05) (Figure 7).

### 3.5. Analysis of Brain Neuropathy Caused by Depression in Patients with ESRD

Depression often leads to the expansion of physical symptoms in patients with cerebral stroke, which generally causes double damage to the normal physical and social functions of patients, and at the same time seriously affects the self-psychological adjustment function of patients. The impact of psychological problems often leads to patients giving up or interrupting treatment, and then, they lose hope for subsequent life and recovery, which directly or indirectly affects the positive cooperation of patients in clinical treatment, thus affecting the best time for rehabilitation of patients and causing serious burdens on families and society (Figure 8). After stimulation of the vagus nerve, the brain activity of patients increased significantly. Patients with severe depression should communicate effectively with the attending physician timely and relieve anxiety and depression as much as possible after using certain antidepressant drugs. Then, further psychological treatment and psychological care were conducted. Figure 8 is a DWI image of the patient's skull. Both T2 and diffusion effects can cause DWI signal enhancement, and lesions with reduced or limited diffusion had higher signals on DWI images. In the imaging process, there was false positive performance with reduced dispersion due to the residual T2 component. Figures 8(a)–8(d) all show the characteristics of clear imaging and high resolution.

The article "Diffusion Tensor Imaging Features of Watershed Segmentation Algorithm for Analysis of the Relationship between Depression and Brain Nerve Function of Patients with End-Stage Renal Disease" was published in 2021. Journal: J Healthc Eng.

## 4. Discussion

ESRD is the end stage of chronic renal failure [15]. It generally refers to the middle and late stages of various types of chronic renal diseases, which is somewhat similar to the concept of uremia, but there are still some differences in the diagnostic criteria. When the chronic renal disease reaches the fifth stage, it enters the end stage of renal disease. At this time, with the further decline of renal function, the patients continue to accumulate toxins in the body, which may cause various symptoms of uremia. The patients generally maintain their normal life through hemodialysis. In addition, if the appropriate renal source can be found for transplantation and replacement, it can be treated. However, the psychological state of patients with such diseases often has various problems, among which depression is the most common [16, 17]. Studies showed that the incidence of depression in ESRD hemodialysis patients is much higher than that in the general population of 20%–30%. Depression is very harmful to hemodialysis patients. Studies indicated that depression in patients before dialysis treatment can produce a series of psychosomatic reactions, increasing the incidence and mortality of cardiovascular diseases [18]. The incidence of depression in ESRD hemodialysis patients was 42.2%, higher than foreign reports. The reasons may be related to the personality and mental stress of Chinese people and factors such as personal tolerance and economic level [19]. The study of Yoong et al. [20] showed that 49.9% of ESRD patients experienced increased depression, and 45.4% of ESRD patients experienced increased anxiety during treatment. The high proportion of anxiety and depression emphasizes the importance of testing and nursing care for ESRD patients during dialysis care. Mu et al. [21] segmented rough semantics in DTI images based on the feature extraction of deep learning, realized super pixel segmentation algorithm, used boundary optimization algorithm to optimize the segmentation accuracy of image edges, and improved the accuracy of image segmentation. In this study, the watershed algorithm was applied to the DWI imaging of patients with brain diseases, which had significant value for the early diagnosis of ESRD patients and psychological care. The correlation analysis of the DTI diffusion index of the segmentation algorithm in the image with the depression score and clinical biochemical indicators. The results showed that the FA value of the anterior left crown was positively correlated with the DST score (*r* = 0.586, *P*=0.007). The FA value of right uppercut was positively correlated with MoCA score (*r* = 0.545, *P*=0.013) and negatively correlated with TMTA (*r* = 0.464, *P*=0.039). The correlation between the results of DTI dispersion index and the blood biochemical indexes of subjects was not significant. The left Nd and subiculum MD values were negatively correlated with depression scores (*r* = −0.463, *P*=0.040).

The article "Diffusion Tensor Imaging Features of Watershed Segmentation Algorithm for Analysis of the Relationship between Depression and Brain Nerve Function of Patients with End-Stage Renal Disease" was published in 2021. Journal: J Healthc Eng.

DTI technology is one of the most effective tools for noninvasively studying the structural and pathological changes of white matter (WM) at the microstructure level. It uses the diffusion anisotropy of water molecules in human tissues, uses various parameters to reflect the direction and degree of water molecule movement in fiber bundles, and visualizes the changes of WM microstructure. The main parameters include the following [22]: fractional anisotropy (FA), axial diffusion coefficient (AD), radial diffusion coefficient (RD), and mean diffusion rate (MD). Moreover, based on the imaging features of watershed segmentation algorithm, ESRD can be diagnosed early. Early treatment can reduce the medical costs, relieve economic pressure, and reduce depression complicated with brain lesions. Asman et al. [23] segmented the medical images and converted the TI-weighted DTI imaging data of the label information of the multiatlas segmentation into fully automated. The segmentation method constructed in the article showed a good effect on the FA of the measured image.

In this study, DTI technology is used to explore the correlation between depression and brain neuropathy in ESRD patients based on methods. The following conclusions are drawn: early diagnosis of ESRD based on watershed segmentation algorithm is conducive to early treatment and reduce depression and brain lesions in ESRD patients.

## 5. Conclusion

The purpose of this study is to use the watershed algorithm to segment the DTI image of the brain of ESRD patients and further analyze and explore the relationship between depression and brain nerve function of ESRD patients. The original DTI data of all subjects were collected and processed based on the watershed segmentation algorithm, and the results of automatic segmentation were evaluated as DSC = 0.9446, MPA = 0.9352, and IOU = 0.8911. The analysis of DTI images after watershed algorithm segmentation suggested that the WM microstructure of patients had undergone a certain degree of change and atrophy, and three main WM fibers had undergone lesions. However, the research content still has some limitations. This study only focuses on a single imaging diagnosis method, and the number of samples is not large enough. Therefore, it is necessary to increase the number of samples and deepen the further exploration of watershed algorithm. In conclusion, this study can analyze and judge the relationship between depression and brain nerve function in ESRD patients through watershed algorithm, which provides certain data support and theoretical basis for the diagnosis and treatment of depression in ESRD patients. The only shortcoming of this study was that the number of cases was not large and the number of subjects included in the experiment was limited. At a certain time, multiple centers can be used to conduct experiments, and the algorithm dataset training required a lot of data, so follow-up work needed to increase the training dataset and increase the accuracy.

The article "Diffusion Tensor Imaging Features of Watershed Segmentation Algorithm for Analysis of the Relationship between Depression and Brain Nerve Function of Patients with End-Stage Renal Disease" was published in 2021. Journal: J Healthc Eng.

## Figures and Tables

**Figure 1:** Comparison of differences in population data of subjects.

**Figure 2:** Image segmentation process based on improved watershed algorithm.

**Figure 3:** Comparison of blood biochemical indexes between SD group and NSD group of patients.

**Figure 4:** Comparison of watershed segmentation graph and original graph.

**Figure 5:** Comparison of neuropsychological cognitive scores among subjects.

**Figure 6:** Comparison of difference values in DIC measurement of brain volume by ESRD based on voxel brain volume measurement. Red: atrophy; yellow: more severe atrophy.

**Figure 7:** Comparison of condition between depression group and nondepression group.

**Figure 8:** Depression causing brain lesions in patients.

## Data Availability

The data used to support the findings of this study are available from the corresponding author upon request.
